The article "Evaluation and Image Analysis of Enterprise Human Resource Management Based on the Simulated Annealing-Optimized BP Neural Network" was published in 2021. Journal: Comput Intell Neurosci.

# Evaluation and Image Analysis of Enterprise Human Resource Management Based on the Simulated Annealing-Optimized BP Neural Network

**DOI:** 10.1155/2021/3133065

**Published:** 2021-11-06

**Authors:** Bo Zhao, Yuanlin Xu, Jun Cheng

**Affiliations:** ^1^Chengdu Sport University, Chengdu, Sichuan 610041, China; ^2^Business School, Sichuan University, Chengdu, Sichuan 610064, China; ^3^School of Academic Research, Party School of Chengdu Committee, Sichuan, Chengdu 610110, China; ^4^School of Electronic and Information, Guangdong Polytechnic Normal University, Guangzhou 510665, China

## Abstract

With the continuous development of social economy and the intensification of social competition, human resource management plays a more and more important role in the whole resource system. How to give full play to the advantages of human resources has become the key issue of human resource management evaluation. However, the current human resource management evaluation system has some problems, such as poor timeliness, one-sidedness, and subjectivity. Therefore, this paper proposes a BP image neural network optimized based on the simulated annealing algorithm to realize enterprise human resource management evaluation and image analysis. Through the learning of different time series samples, the average weight distribution scheme of main indicators is obtained, in which the average weight proportions of *c*_1_, *c*_2_, *c*_3_, and *c*_4_ are 25.5%, 24.8%, 17.9%, and 31.9%, respectively. In the comprehensive evaluation of enterprise employees, the error between the actual output and expected output is less than 4.5%. The results show that the BP image neural network based on simulated annealing algorithm has high accuracy in the image analysis and evaluation of enterprise human resource management. The output analysis results meet the actual needs of the enterprise and the personal development of employees and provide a decision-making scheme for the evaluation of enterprise human resource management.

## 1. Introduction

With China's economy entering the new normal, the traditional extensive enterprise management model has been difficult to meet the needs of the rapid development of social economy. In this context, a large number of traditional enterprises began to change the human resource management mode to refinement. How to realize the matching between personnel and posts and how to formulate scientific human resource planning are the key issues of enterprise human resource reform. The traditional enterprise talent evaluation mainly depends on the experience of experts. This subjective talent evaluation system will have great differences due to different evaluation personnel, and it is difficult to realize the reasonable matching between personnel distribution and the actual work needs of the enterprise, which will eventually reduce the enthusiasm of employees and limit the development of the enterprise. Therefore, building an image analysis and evaluation system of enterprise talent management more in line with the actual needs of enterprises is of great significance to the development and reform of the enterprise human resource management mode.

The article "Evaluation and Image Analysis of Enterprise Human Resource Management Based on the Simulated Annealing-Optimized BP Neural Network" was published in 2021. Journal: Comput Intell Neurosci.

With the significant growth of social informatization, the theory and application of the BP neural network (BP) have made great progress and development and have a far-reaching impact on various fields. Many fields of comprehensive image analysis and evaluation have completed the development and reform of the traditional evaluation model by introducing the new idea of neural network [1]. In the traditional talent evaluation process, the evaluation results are closely related to the experience of evaluation experts. The more experienced the image analysis and evaluation personnel are, the more sensitive they are to data information processing and the closer the final evaluation result is to the actual value. The evaluation process is very consistent with the working principle of the BP neural network [2]. It is feasible to introduce the BP neural network into the talent evaluation system. The introduction of the BP neural network can reduce the subjective judgment error, make the enterprise human resource management system more objective and the evaluation results more scientific and reasonable, and provide the most appropriate countermeasures and suggestions for the long-term development of enterprises and the application of single materials. However, the traditional BP neural network image analysis has some problems, such as slow convergence speed, high sensitivity to weight initialization, and easy to fall into the local extremum, which affect the accuracy and rationality of the evaluation results [3].

In order to solve the problems of large subjective judgment error, slow convergence speed, and easy to fall into the local extremum in the traditional enterprise human resource management mode when the existing BP neural network is used for talent evaluation, this paper proposes a talent analysis and evaluation model based on simulated annealing algorithm in order to achieve an objective, scientific, and reasonable output. The BP image neural network optimized by simulated annealing algorithm is proposed in this paper to realize the evaluation and image analysis of enterprise human resource management. The innovative contribution of this paper is to train the BP neural network model with low temperature and fast cooling speed by using simulated annealing (SA) algorithm, which effectively avoids the weight and deviation of the BP neural network falling into the local extreme value and provides a new optimization scheme for the reform of the enterprise human resource management mode. The algorithm in this paper solves the shortcomings of traditional BP neural network image analysis. It has the advantages of fast convergence speed, low sensitivity to weight initialization, and not easy to fall into the local extremum, and it can measure and evaluate the results more accurately and reasonably.

The article "Evaluation and Image Analysis of Enterprise Human Resource Management Based on the Simulated Annealing-Optimized BP Neural Network" was published in 2021. Journal: Comput Intell Neurosci.

Section 1 briefly introduces the research background and significance of enterprise human resource management evaluation.  Section 2 briefly introduces the research status of enterprise human resource management evaluation, discusses the existing problems in this field, and summarizes the research work and research methods of this paper.  Section 3 introduces the image analysis process of the BP neural network optimized by simulated annealing algorithm and studies the evaluation of enterprise human resource management based on the SA-BP (simulated annealing-backpropagation) neural network model.  Section 4 establishes the evaluation index of enterprise human resource management, trains and tests the SA-BP neural network, and finally analyzes the output of the network.  Section 5 is a brief summary of the main conclusions.

## 2. Related Work

Many scholars have done a lot of work on the evaluation method of human resource management. Fowler et al. put forward the need to carry out research on human resource soft management as early as 1992 [4]. Coutinho et al. developed the human resource utility index using the data of the human resource management system to evaluate the effectiveness of human resource management [5]. Ming et al. evaluated human resource management through the organizational health report index [6]. Lappan and Brain Towers proposed the human resource scorecard to realize the comprehensive consideration of human resource strategy, operation, customer, and finance [7]. Loyarte Lopez et al. proposed the personnel maturity model to help enterprises find the advantages and disadvantages of personnel management [8]. Chen et al. proposed the quality evaluation model of human resource management from the perspective of personnel maturity and put forward the key time and standard business process that constitute the KPA [9]. Boudlaie et al. believed that the human resource scorecard proposed by Brian E. Beeker only stayed at the level of theoretical research and built the human resource management efficiency scorecard on this basis, which increased the operability of the human resource scorecard from four aspects of human resource strategy, operation, customer, and finance [10]. Zhang and Jing analyzed the core ideas and indicators of the four aspects in the scorecard and included all employees in the scope of assessment and evaluation [11]. All of these methods are localized research based on foreign evaluation methods.

The article "Evaluation and Image Analysis of Enterprise Human Resource Management Based on the Simulated Annealing-Optimized BP Neural Network" was published in 2021. Journal: Comput Intell Neurosci.

Domestic scholars have also done a lot of work in the evaluation of human resource management by establishing the index system. Rajesh and Rajendran divided the practice process of human resource management into four parts: recruitment, training, performance evaluation, and incentive. However, these contents still remain in the traditional personnel management function and cannot make a basic prediction of the future supply and demand of human resources [12]. To this end, Klimecka-Tatar and Ingaldi added two indicators of human resource planning and information management on the basis of the original index system [13]. Wei and Jin proposed the research on the performance evaluation and optimization of human resource management based on BP algorithm, introduced the artificial neural network into the evaluation of human resource management, established the evaluation model of human resource management based on BP algorithm, and put forward countermeasures [14]. Chen and Tian proposed a quantitative evaluation method of human resource management based on Markov analysis and established a quantitative model to evaluate the advantages and disadvantages of human resource management methods by using Markov analysis [15].

To sum up, although many scholars have done a lot of research work in enterprise human resource evaluation, the one-sidedness and subjectivity of evaluation methods based on organizational science have become an important factor restricting the development of human resource evaluation methods. Therefore, how to make the evaluation method objective and fair is an urgent problem to be solved in the research of enterprise human resource management evaluation. Although the introduction of the BP neural network provides a new idea for the improvement of the human resource image evaluation model, the traditional BP neural network has some problems, such as slow convergence speed, sensitive to weight initialization, and easy to fall into the local extremum, which also affect the accuracy and rationality of image evaluation results. In view of this, the BP neural network model based on simulated annealing algorithm proposed in this paper can solve the problems of slow convergence and easy to fall into the local optimal solution and realize an objective, scientific, and reasonable evaluation method.

The article "Evaluation and Image Analysis of Enterprise Human Resource Management Based on the Simulated Annealing-Optimized BP Neural Network" was published in 2021. Journal: Comput Intell Neurosci.

## 3. Image Evaluation Model of Human Resource Management Based on the Simulated Annealing-Optimized BP Neural Network

### 3.1. Optimization of the BP Neural Network Image Model Based on the Simulated Annealing Algorithm

BP neural network is a multilayer feedforward neural network trained according to the error backpropagation algorithm, which can complete the algorithm model of nonlinear mapping [16]. In the setting of the BP neural network, the number of input and output layer neurons, the number of hidden layer neurons, the learning rate, and the selection of transfer function are considered. Its general structure is shown in Figure 1.

It can be seen from Figure 1 that the external information is input from the input layer and transferred to the hidden layer through the BP neural network. In the hidden layer, the transfer function and weight information are combined to reclassify and sort. The minimum transmission distance between neurons can be expressed as

(1) $$\begin{array}{c} P\left(x\right)=\left|A_{x}-B_{x}\right|=\sqrt{\sum_{x=1}^{n}{\left[A_{x}-B_{x}\right]}^{2}}. \end{array}$$

In formula (1), *n* is the number of neurons; *A*_*x*_ is the weight of neuron *x*; *B*_*x*_ is the output value of neuron *x*. The smaller the value of *P*(*x*), the higher the similarity between *A*_*x*_ and *B*_*x*_.

In the BP neural network, if there are too many information nodes in the hidden layer, the effective information to be processed will also increase, which will lead to too long training time of the model and even overfitting phenomenon. Therefore, reasonable selection of the number of hidden layers and neurons is the key to the construction of the BP neural network. The optimal number of hidden layer nodes can be obtained by the following formula:

(2) $$\begin{array}{c} H_{x}=\frac{\sum_{x=1}^{n}\left(S_{x}-T_{x}\right)}{P\left(x\right)}. \end{array}$$

In (2), *H*_*x*_ is the optimal number of nodes in the hidden layer; under this node, the best training time can be obtained by calculation, and the efficiency *S*_*x*_ and accuracy *T*_*x*_ of the neural network will be in the best state.

From the output layer to the hidden layer, the weight of the BP neural network is adjusted in the direction of reducing the error according to certain principles:

(3) $$\begin{array}{c} \alpha_{e}=\left[P_{e}\left(\Delta x\right)-H_{e}\left(\Delta x\right)\right]\cdot f\left(e\right). \end{array}$$

In (3), *f*(*e*) is the connection weight between two nodes, *P*_*e*_ is the connection weight along the *e*-direction, and Δ*x* is the weight change. The total connection weight of each neuron receiving information input from other neurons can be expressed as

(4) $$\begin{array}{c} W_{ij}=\int_{i=1}^{n}\left[k_{ij}x_{i}+\alpha_{e}\left(i\right)\right]. \end{array}$$

In formula (4), *W*_*ij*_ is the binding strength of neurons *i* and *j*, which is the connection weight; *x*_*i*_ is the output of the neuron; *α*_*e*_(*i*) is the threshold of neuron *i*. In order to make the network accurate and reliable, it is necessary to ensure that the output value of the network and the expected value are within a certain range, and this evaluation index is generally expressed by the sum of squares of errors *E*, and its mathematical expression is as follows:

(5) $$\begin{array}{c} E=\frac{1}{u}\cdot \sum_{i=1}^{n}\sum_{j=1}^{m}r{\left[W_{ij}-\bar{W_{ij}}\right]}^{2}. \end{array}$$

In equation (5), *u* is the number of neurons in the hidden layer, *m* is the number of neurons in the input layer, *n* is the number of neurons in the output layer, and *r* is a random constant from 1 to 10. The general range of the number of neurons can be determined by the calculation of the above formula, and the optimal number of neurons in the hidden layer can be determined by selecting the intermediate value.

The article "Evaluation and Image Analysis of Enterprise Human Resource Management Based on the Simulated Annealing-Optimized BP Neural Network" was published in 2021. Journal: Comput Intell Neurosci.

After determining the number of hidden layers and neurons, we need to know the threshold *k*_*i*_ between the hidden layer and the output layer. When the output value of the *i* neuron in the hidden layer is *y*_*i*_, the expression is as follows:

(6) $$\begin{array}{c} y_{i}=\int_{i=1}^{n}k_{i}\left(ld_{i}-bu_{i}\right). \end{array}$$

In (6), *d*_*i*_ is the connection weight between the input layer node and the hidden layer node; *u*_*i*_ is the connection weight between the hidden layer node and the output layer node; *I* is the expected output value; *b* is the error value of weight. The error function is usually chosen as the evaluation index of the BP neural network:

(7) $$\begin{array}{c} U_{ij}=\frac{1}{mn}\sum_{i=1}^{m}\sum_{j=1}^{n}{\left(\rho_{ij}-\sigma_{ij}\right)}^{2}. \end{array}$$

In equation (7), *m* is the number of training samples; *n* is the number of neurons in the output layer; *ρ* is the expected output value; *σ* is the actual output value.

As a self-learning neural network model, BP neural network adjusts the weight of nodes according to the error between the actual output value and the expected output value of neurons:

(8) $$\begin{array}{c} y_{ij}=\alpha U_{ij}+\beta W_{ij}+\gamma E_{ij}. \end{array}$$

In (8), *y*_*ij*_ is the weight between input neuron *i* and regular neuron *j*.

(9) $$\begin{array}{c} Y_{ij}=1+c{\left(\frac{y_{ij}}{\alpha_{ij}}-\frac{y_{ij}}{\beta_{ij}}-\frac{y_{ij}}{\gamma_{ij}}\right)}^{2}. \end{array}$$

In (9), *α*_*ij*_ and *β*_*ij*_ are the evaluation scores of forward transmission and backward transmission, respectively.

The article "Evaluation and Image Analysis of Enterprise Human Resource Management Based on the Simulated Annealing-Optimized BP Neural Network" was published in 2021. Journal: Comput Intell Neurosci.

Through the training of a certain number of samples, the appropriate weight parameters of the network can be determined; thus, in the case of *n* sample inputs, the residual value between the actual output *o* and *o'* is minimized to

(10) $$\begin{array}{c} Q_{t}=\frac{1}{2}\sum_{i,j=1}^{n}\frac{Y_{ij}}{t}. \end{array}$$

In equation (10), *t* is the number of iterative corrections, and the reasonable weights and control parameters of the model can be determined by the backpropagation gradient method. After the construction and training of the BP neural network, in order to solve the problems of low convergence speed and easy to fall into the local extremum, the cooperative algorithm model of simulated annealing algorithm and BP neural network is established. The algorithm flowchart is shown in Figure 2.

As can be seen from Figure 2, the BP neural network optimized by simulated annealing algorithm is mainly divided into four parts: constructing the BP model, randomly setting the weight of each neuron, using simulated annealing algorithm to obtain the optimal weight and deviation, and judging the termination of training [17]. After determining the above steps, it is necessary to consider the selection of initial temperature, temperature attenuation function, and end condition, in which the Boltzmann annealing function is usually selected as the temperature attenuation function, and its mathematical expression is as follows [18]:

(11) $$\begin{array}{c} F\left(\text{state}\right)\infty e^{-\left(E/kT\right)}. \end{array}$$

In (11), *E* is the state energy; *kT* is the product of Boltzmann constant and thermodynamic temperature. The ratio of Boltzmann distribution between two states of a system is called Boltzmann factor:

(12) $$\begin{array}{c} \frac{F\left(\text{state }2\right)}{F\left(\text{state }1\right)}=e^{E_{1}-E_{2}/kT}. \end{array}$$

The general form of the neural network is as follows:

(13) $$\begin{array}{c} \text{net}=w^{T}x+b. \end{array}$$

For the output vector *Y* of a neuron, it can only be taken as 0 or 1. If *Y* = 1, then the probability is *p*:

(14) $$\begin{array}{c} P\left\{Y=1|x\right\}=p\left(x\right)=\frac{1}{1+e^{-\left(\text{net}/T\right)}}. \end{array}$$

If *Y* = 0, the probability is *1* − *P* and then changes to

(15) $$\begin{array}{c} P\left\{Y=0|x\right\}=p\left(x\right)=\frac{1}{1+e^{net/T}}. \end{array}$$

Then, the system transition probability here is

(16) $$\begin{array}{c} \frac{P\left\{Y=0|x\right\}}{P\left\{Y=0|x\right\}}=\frac{p\left(x\right)}{1-p\left(x\right)}=e^{\text{net}/T}. \end{array}$$

Equation (16) is the Boltzmann factor of the Boltzmann temperature decay function. The key of simulated annealing algorithm is the cooling process, and if the cooling process is too fast, the global optimal solution will be lost; too slow will increase the execution time of the algorithm. Therefore, the selection of an appropriate temperature decay function is of great significance to the optimization performance of simulated annealing algorithm [19].

The article "Evaluation and Image Analysis of Enterprise Human Resource Management Based on the Simulated Annealing-Optimized BP Neural Network" was published in 2021. Journal: Comput Intell Neurosci.

### 3.2. Image Evaluation of Enterprise Human Resource Management Based on the SA-BP Model

A reasonable enterprise human resource management scheme is not only in line with the actual needs of enterprise personnel but also meets the personal development [20]. Therefore, in view of the strong subjectivity of the existing enterprise human resource management evaluation mode and the greater influence of experience, this paper studies and proposes the SA-BP model to realize the reasonable and scientific evaluation of enterprise personnel, and its specific implementation process is shown in Figure 3.

As can be seen from Figure 3, the first step of enterprise human resource management evaluation research needs to analyze the factors affecting enterprise human resource management evaluation, establish evaluation indicators, refine and quantify indicators, and form a system; secondly, it is necessary to establish the SA-BP neural network, including the determination of the network layer, the number of neurons in each layer, learning rate, and initial value [21]. Then, the neural network is trained and tested by using the index data of image quantization, and the network converges through continuous iterative correction. Finally, the quantitative indexes of employees are input into the trained SA-BP neural network model to obtain the comprehensive evaluation score.

## 4. Application Effect Image Research of the SA-BP Neural Network Optimized by the Simulated Annealing Algorithm

### 4.1. Determination of the Human Resource Management Evaluation Index

This paper studies and constructs an enterprise human resource management evaluation index system with 4 first-level indexes and 10 second-level indexes. Among them, the first-level indicators are individual function *c*_1_, work experience *c*_2_, work ability *c*_3_ and theoretical knowledge *c*_4_ [22]. In order to make the division of different types of indicators more scientific, the correlation analysis of *c*_1_, *c*_2_, *c*_3_, and *c*_4_ variables was carried out.

As shown in Figure 4, the correlation between *c*_1_, *c*_2_, *c*_3_, and *c*_4_ is low, which has obvious differentiation as an enterprise human resource evaluation index. The secondary indicators include age *a*_1_, gender *a*_2_, length of service *a*_3_, postage *a*_4_, department age *a*_5_, vocational qualification level *a*_6_, professional and technical level *a*_*7*_, expert talent type *a*_8_, graduate school *a*_9_, and academic level *a*_10_ [22]. The correlation analysis of the secondary indicators is carried out.

The article "Evaluation and Image Analysis of Enterprise Human Resource Management Based on the Simulated Annealing-Optimized BP Neural Network" was published in 2021. Journal: Comput Intell Neurosci.

As can be seen from Figure 5, except for the strong correlation between postage and working age, the correlation coefficients of other secondary indicators are all below 0.5, indicating that the correlation between the indicators is weak, and there is no significant linear relationship, so it can contain more abundant evaluation information when reflecting the weight of primary indicators.

### 4.2. Training and Testing of the SA-BP Neural Network

The quality of training data directly affects the output of the neural network model. According to the determined primary and secondary indicators, in order to consider the impact of time series, four groups of evaluation objects in different years are selected, and their indicators are quantified [23]. The index data of the image evaluation object are normalized to obtain the learning sample input of the SA-BP neural network. At the same time, the comprehensive score of the evaluation object is output as a learning sample by the entropy method [24]. The evaluation results of the neural network trained by this image method are not only in line with the expert evaluation system but also in line with the actual needs of enterprises. Through the learning and training of four groups of different time series samples, SA-BP neural network gives the weight relationship of each group's human resource management evaluation index, as shown in Figure 6.

It can be seen from Figure 6 that the weights of the first-level indicators of the networks trained by different time series learning samples are very different, and the weight of individual physical fitness accounts for 48% of the total in the first year; in the second year, the weight of work ability accounted for 37.1%; in the third year, work experience accounted for 39.5%; in the fourth year, work experience accounted for 38.4%. The results show that the evaluation of human resource management based on expert experience is very subjective. In order to make the network more objective and scientific, the weight distribution of the first-level indicators in four years is averaged on the basis of expert experience. The average weight distribution of the first-level indicators is shown in Figure 7.

It can be seen from Figure 7 that theoretical knowledge has the greatest impact on the final evaluation results, accounting for 31.87%; in addition, the weight proportion of personal physique, work experience, and work ability decreased, which was 25.47%, 24.78%, and 17.88%, respectively. The assignment scheme is used as the main index weight assignment scheme of the neural network. At the same time, the neural network trained by learning sample set needs image testing. The test sample set is obtained through a questionnaire survey of 16 enterprise employees. Like the test set images, in order to make the analysis results more scientific, it is necessary to standardize the original data [25]. After training, the SA-BP neural network is tested by image, and the results are shown in Figure 8.

The article "Evaluation and Image Analysis of Enterprise Human Resource Management Based on the Simulated Annealing-Optimized BP Neural Network" was published in 2021. Journal: Comput Intell Neurosci.

It can be seen from Figure 8 that the error between the actual output and the expected output of the network can be controlled within 4.5%, indicating that the trained SA-BP neural network has good evaluation results, which can be used for the follow-up study of enterprise human resource management evaluation.

### 4.3. Output Analysis of the SA-BP Neural Network

Using the trained SA-BP neural network, according to the corresponding quantitative index, 10 employees are evaluated comprehensively. The network output is shown in Figure 9.

It can be seen from Figure 9 that the actual output results of the trained SA-BP neural network are basically consistent with the results obtained by the entropy method. The results show that the use of neural network evaluation can not only meet the output results consistent with expert experience but also make the evaluation system objective and quantitative, so as to realize the scientific and reasonable evaluation of human resource management. The relationship between the actual output and the ideal output is better quantified by bit, and the output error of the drawing network is shown in Figure 10.

It can be seen from Figure 10 that the output error of the model is within 4.5%, and the actual evaluation score is close to the evaluation score given by expert experience. The results show that the output results of the BP neural network based on simulated annealing algorithm not only accord with the experts' evaluation experience but also can be scientific, objective, and fair to the greatest extent. It can not only meet the actual needs of the enterprise but also give full play to the strengths of each employee, which can be used as the evaluation basis of enterprise human resource management.

## 5. Conclusion

Aiming at the problems of strong subjectivity and unreasonable allocation of personnel and posts in the evaluation of traditional enterprise human resource management, this paper proposes a BP image neural network optimized by simulated annealing algorithm to realize the evaluation and image analysis of enterprise human resource management. This paper introduces the image analysis process of the BP neural network optimized by simulated annealing algorithm and studies the evaluation of enterprise human resource management based on the SA-BP (simulated annealing-backpropagation) neural network model. At the same time, the evaluation index of enterprise human resource management is established, the SA-BP neural network is trained and tested, and finally, the output of the network is analyzed. Through the learning of different time series samples, the average weight distribution scheme of main indicators is obtained. The results show that the algorithm solves the shortcomings of traditional BP neural network image analysis. The algorithm has the advantages of fast convergence speed, low sensitivity to weight initialization, and not easy to fall into the local extremum. It can measure and evaluate the results more accurately and reasonably. The contribution of this paper is to train the BP neural network model with low temperature and fast cooling speed by using simulated annealing (SA) algorithm, which effectively avoids the weight and deviation of the BP neural network falling into the local extreme value and provides a new optimization scheme for the reform of the enterprise human resource management mode. Since the data of the proposed scheme are not verified in this paper, it needs to be further optimized in future research.

The article "Evaluation and Image Analysis of Enterprise Human Resource Management Based on the Simulated Annealing-Optimized BP Neural Network" was published in 2021. Journal: Comput Intell Neurosci.

## Figures and Tables

**Figure 1:** Structure distribution of the BP neural network model.

**Figure 2:** Flowchart of the BP neural network algorithm based on simulated annealing algorithm optimization.

**Figure 3:** Evaluation model of enterprise human resource management based on the SA-BP neural network.

**Figure 4:** Correlation analysis of primary indicators.

**Figure 5:** Correlation analysis of secondary indicators.

**Figure 6:** Weight distribution of the first-level indicators of human resource management evaluation in enterprises with different learning samples.

**Figure 7:** The average weight distribution of the first-level index of enterprise human resource management evaluation.

**Figure 8:** SA-BP neural network test sample error.

**Figure 9:** Output results of the SA-BP neural network.

**Figure 10:** Output error of the SA-BP neural network.

## Data Availability

The data used to support the findings of this study are available from the corresponding author upon request.
